# The Effect of Comprehensive Rehabilitation Nursing on the Rehabilitation of Sports-Induced Ankle Joint Injuries

This article has been retracted.

**DOI:** 10.1155/2022/4004965

**Published:** 2022-05-24

**Authors:** Yu Qiao, Bin Zhang, Lei Zhang

**Affiliations:** ^1^Angeles University Foundation, Angeles City, Pampanga, Philippines; ^2^Anhui Normal University, Wuhu 241000, Anhui, China; ^3^Anhui Wannan Medical College, Wuhu 241000, Anhui, China

## Abstract

The purpose of participating in sports is to enhance physical fitness and promote physical and mental health. The occurrence of sports injuries will cause physical and mental injuries to athletes, especially the ankle joint injuries that often occur. Therefore, it is particularly important to understand the causes, symptoms, treatment, and prevention of athletes' ankle injuries. This article aims at studying the significance of comprehensive rehabilitation nursing for the rehabilitation of sports-induced ankle joint injuries and introduces the concepts of comprehensive rehabilitation nursing and ankle joint injuries. This article proposes how to use comprehensive rehabilitation nursing to recover ankle injuries caused by sports based on smart medical care. In the experiment of this article, it can be seen from Table 5 that the recovery speed of 5 athletes with ankle joint injuries before rehabilitation training was 8% (lowest) and 14% (highest). The recovery rate after rehabilitation care is up to 25%. It can be seen that comprehensive rehabilitation care is of great help to athletes with ankle injuries. As can be seen from Table 4, the number of ankle injuries in acute secondary injuries is 25, accounting for 33%, which is the highest; the number of contusions is 15, accounting for 21%, which is the lowest ratio, so it can be seen that the ankle joint injury in sports is the most serious. Therefore, the application of comprehensive rehabilitation care needs to be popularized, which is of great significance to ankle joint injuries. The ankle joint is one of the most easily sprained joints in the human body, not only because of the flexibility of the ankle joint, but also because of the anatomical characteristics of the ankle joint. The main cause of ankle injuries is inappropriate behavior in sports.

## 1. Introduction

Ankle joint injuries mainly include fractures of the ankle joint and damage to the surrounding ligaments. This is a relatively common sports injury. If an ankle joint injury occurs without timely and effective treatment or without thorough treatment, it will be easier to cause repeated attacks in the future, and it is not easy to recover. With the development of the national economy, the advancement of modern science, and technology and the improvement of people's living standards, the importance of rehabilitation medicine is increasingly recognized by people. Even in some foreign countries with advanced science, rehabilitation medicine is a relatively new discipline, and rehabilitation nursing must gradually form an independent system from nursing and become a new field of nursing [1].

The ankle joint injuries of students majoring in physical education are increasing year by year during the learning process. More and more educators are beginning to pay attention to ankle injuries and rehabilitation training after injuries. Improving students' awareness of their own protection is the main purpose. Due to the structure of the human body and the physiological characteristics of the ankle joint, students will suffer more injuries during the learning process. Making a reasonable and effective rehabilitation plan based on injury symptoms is a method of rehabilitation, and how to deal with ankle joint injuries is a problem that needs to be solved urgently.

Over the years, with the development of social economy and the change of cultural structure, the country has paid more and more attention to sports. Kai found that ankle ligament injuries often occur in sports, and the most common injuries include hands and feet. In general, conservative treatment is the first choice of treatment. The increasing severity of athletes' long-term injuries and the associated expensive treatment costs indicate that ankle joint injuries should not be underestimated. The scholar argued that ankle joint injuries should not be ignored, but there is a lack of data and authenticity [2]. Besting A found that due to supplier independence, new Internet service-oriented points of care and surgical equipment are the basis for improved operations. In order to improve efficiency, people should actively develop new methods. In this work, scholars discuss how to deal with these challenges and develop a descriptive model to determine key strategies. But the experiment did not mention what the new method is, and the concept is too vague [3]. Lacey and Donne found that ankle joint injuries not only lead to the destruction of static and dynamic balance, but also result in wasting a lot of exercise time, affecting athletes' daily activities, and may put athletes at greater risk of injury. Therefore, in order to identify athletes at risk of ankle injury, accurate and reliable balance assessment tools are needed. The balance test they proposed has strong reliability. The disadvantage of this experiment is that there is no experiment on the balance of the method, so the reliability cannot be confirmed [4]. Acosta-Olivo et al. found that overweight can also cause some injuries during sports. The purpose of his research is to assess whether there is a link between acute ankle injury and body mass index. But through experiments, they finally found that obesity is not a factor that affects ankle joint injury, and age is the key determinant of ankle joint injury. The disadvantage of this experiment is that it directly draws a conclusion. There is no object reference and process for the experiment, which makes the experiment very incomplete [5]. Lo et al. found that the mobile medical information system has a great impact on the traditional hospital information system, and the dynamic resource allocation table is very important for optimizing the performance of the mobile system. He designed an intelligent dynamic resource allocation model, using algorithms and cumulative allocation to optimize the resource allocation weights of the five main attributes in the cooperative communication system. Finally, it is found that the designed model can improve the efficiency of the medical system. This method does not propose what the specific model is and how the model is designed [6]. Ghoneim et al. found that with the invention of new communication technologies, artificial intelligence provides new functions and facilities for the smart medical framework. These functions and facilities are designed to provide customers with seamless, easy-to-use, accurate, and real-time healthcare services. Since health is a sensitive issue, it should be treated with the utmost safety and caution. The experiment did not compare artificial intelligence with traditional methods and did not compare the advantages of artificial intelligence [7]. Rana and Mishra found that the smart health medical system can not only improve the quality of medical services, but also improve the security of the system. The original system will have the problem of data insecurity and privacy insecurity in the smart health system. In order to overcome security and privacy risks, they designed effective access control for medical services. However, the program has not been proven, and no effective experiments are provided to solve [8]. Tian et al. found that with the development of information technology, smart medical care makes medical treatment more efficient, more convenient, and more personalized. In order to introduce the concept of smart medicine, Tian et al. first introduced the current situation of smart medicine in several important areas. Finally, they look to the future and evaluate the future prospects of smart medicine. Although they saw the advantages of artificial intelligence, they did not see the shortcomings of artificial intelligence and did not consider the pros and cons between the two [9]. Through the experimental analysis of scholars, we can see that as the field of sports expands, more and more people love sports. However, due to many factors, more and more people are causing ankle injuries. So scholars have conducted experiments on ankle joint injuries.

The innovations of this article are as follows: (1) introduced the relevant theoretical knowledge of smart medical treatment and ankle joint injury, and used data mining to analyze how comprehensive rehabilitation care plays a role in the rehabilitation of ankle joint injury, and (2) analyzed the data fusion, and conducted experiments and analysis on the injury factors and preventive measures of the ankle joint. Through experiments, it has been found that the proportion of ankle joint injuries has increased in recent years. There are many factors affecting the ankle joint. How to prevent ankle joints and use comprehensive rehabilitation care to recover ankle joint injuries is of great significance.

## 2. Data Mining Method and Multisource Data Fusion Algorithm Based on Smart Medical Care

Smart healthcare is a new term in medical care. By building a regional medical information platform for health records and using the most advanced Internet of Things technology, the interaction between patients and medical personnel, medical institutions, and medical equipment can be realized gradually, and information is gradually achieved [10, 11]. Ankle injuries are the most common sports injuries. It is mainly caused by the changes in the force acting position, direction, size, and other factors, as well as the different movement status of the lower limbs [12]. The degree of injury and the shape of the ankle joint are different, so the mechanism of the ankle joint injury is extremely complex and diverse.

The human body model uses high-resolution CT scanning to digitize the anatomical structure of the human body and is divided into fine finite element meshes to accurately simulate the geometric structure of the human body. The model reflects the anatomical characteristics of each organ. It can simulate damage at the tissue level by inputting the data of the physical material properties of organs and tissues reported in the latest research [13]. Simulated ankle injury is shown in Figure 1.

As shown in Figure 1, the reasons for ankle joint injury during exercise are not being prepared for exercise before exercise, the muscles and ligaments of the ankle not being open, and the elasticity and stretchability of the joint ligaments being poor and not able to adapt to the needs of strenuous exercise [14].

### 2.1. Multisource Data Fusion Based on Smart Medical Care

The configuration of multisensor systems in medical care provides necessary conditions for the application of multisource data fusion. Multisource data fusion technology can realize applications such as behavior monitoring based on motion information and medical diagnosis based on physiological information by using the information collected by multisource sensors in smart medical care [15, 16]. Data-level fusion, also called pixel-level fusion, is a low-level fusion. After collecting the data, the sensor only performs simple processing or starts data fusion without processing. On the basis of the fusion, the characteristic information is extracted to obtain the final result. Data-level fusion generally requires the data collected by the sensor to be the same physical quantity. This level of fusion retains as much information as possible during the calculation process, and the fusion accuracy is the highest, but it is also accompanied by a large amount of calculation and a slow calculation speed [17].

The level of multisource data fusion is different, and the algorithms used are also quite different. Methods such as weighted average Kalman filtering are generally applied to low-level fusion. In high-level fusion, methods such as evidence theory, neural networks, and Bayesian inference are often used. Different levels of integration have their own advantages and disadvantages, and should be applied according to specific requirements. Choose an appropriate method to process the data at a specific level to achieve the best results [18]. The structure of multisource data fusion is shown in Figure 2.

As shown in Figure 2, according to the actual situation and application requirements of the obtained data, a certain degree of preprocessing is carried out on the data. Including inconsistency elimination, filling in missing data, and data standardization operations, the preprocessed data have higher quality [19]. Although the DS evidence theory can effectively deal with uncertain information, in the case of highly conflicting evidence, the classical DS evidence combination rules often produce unreasonable fusion results due to the normalization process. For this reason, many scholars have proposed many differences. Based on the modified method, the evidence distance is introduced, and the feature extraction of the evidence source is carried out, and the corresponding improvement scheme is put forward. The theoretical analysis and numerical experimental results show that the improved method can not only fully reflect the corresponding improvement ideas, but also can better realize the evidence combination, converge the real target faster, and get a reasonable fusion result.

Fusion computing is the use of one or more multisource data fusion algorithms to complete the fusion processing of feature data. Feature extraction and fusion calculation are the core of the entire fusion process. According to the data obtained by the fusion calculation, through certain decision rules, the final decision result is obtained for output. infusion computing is shown in Figure 3.

As shown in Figure 3, for data-level fusion with a lower fusion level, in order to retain more detailed information of the original data, there is often no data preprocessing link. In data processing, first go through fusion calculation and then extract features on the basis of the fusion result to obtain the final result [20].

#### 2.1.1. Evidence Theory

Based on the historical data provided by the smart medical database and the rule method provided by the knowledge base, the system determines to adopt the membership function to obtain the initial credibility of the evidence theory. Membership function, also known as the membership function or fuzzy meta-function, is a function that will be used in fuzzy sets and is a generalization of indicator functions in general sets. An indicator function can tell whether an element in a collection belongs to a particular subcollection. The basic reliability distribution of the data to be tested in different physical states is given as

(1) $$\begin{array}{c} A_{i}=\frac{1}{e^{\left(u/\sigma^{2}\right)}},\;u=1,2,3, \end{array}$$

where *e*^(*u*/*σ*^2^)^ and *A*_*i*_ correspond to the historical data about body temperature provided by the database in the u-th physical sign state.

Through the combination of the evidence theory, the evidence is merged, and the reliability matrix *H* is obtained as

(2) $$\begin{array}{c} H=\left(H_{A},H_{B},H_{C}\right). \end{array}$$

Evidence theory is widely used to solve uncertain reasoning problems, and it is an important data processing method for multisource data fusion. For an evidence theory problem model, all possible results are included in the identification framework Θ. The evidence theory uses sets to represent propositions, and Θ represents the set containing all the results of a problem. That is, Θ={*θ*_1_, *θ*_2_,…, *θ*_*n*_}, where *θ*_*n*_ is called an element in the recognition frame, and different elements are mutually exclusive [21].

The reliability function is the main mathematical tool to describe the subjective uncertain phenomenon. The main difference between the reliability function and the probability function is that it does not satisfy the additivity. More importantly, there is Dempster's rule in the theory of reliability function, which can be used to combine two independent reliability functions into a comprehensive reliability function. The basic reliability function is used to express the degree of people's trust in the evidence. Suppose the recognition framework is Θ, and the basic reliability function is

(3) $$\begin{array}{c} \left\{\begin{array}{c} m\left(\varphi \right)=0,\\ \sum_{A\subseteq 2^{\Theta }}m\left(A\right)=1, \end{array}\right. \end{array}$$

where *m*(*φ*)=0 means that the empty set does not have any reliability. For any subset A, as long as it satisfies *m*(*φ*)≻0, A is called a focal element.

How to merge the evidence is the key of the evidence theory algorithm, and this method is also called the D-S synthesis rule. Assuming that *m*_1_ and *m*_2_ are the basic reliability functions in the recognition framework Θ, the D-S synthesis rule is

(4) $$\begin{array}{c} m\left(A\right)=\frac{1}{1-k}\sum_{a\cap b}m_{1}\left(A_{i}\right)m_{2}\left(B_{J}\right), \end{array}$$

where *m*_2_(*B*_*J*_) is the conflict coefficient, and its size is between 0 and 1, indicating the degree of conflict between evidence. The larger the *K*, the higher the degree of conflict between the evidence.

Evidence theory can effectively distinguish “unknown” and “uncertain” information. And compared with the Bayesian theory in the probability theory, the evidence theory does not need to obtain conditions such as prior probability and conditional probability density, and has obvious advantages in dealing with uncertainty problems [22].

#### 2.1.2. Improved Evidence Theory

Because the prior data required in the theory of evidence are more intuitive and easier to obtain than those in the theory of probabilistic reasoning, with its own advantages, the evidence theory has played a huge role in solving related problems of uncertain reasoning and has become a basic algorithm in the field of data fusion [23]. However, its theory also has some problems, such as strict requirements on combination conditions, and each piece of evidence must be independent of each other.

Some scholars start by modifying the initial evidence reliability model, averaging the basic reliability values of different evidences, and then synthesize them with the D-S synthesis formula. The method of obtaining new evidence is

(5) $$\begin{array}{c} m\left(A\right)=\frac{1}{n}\left(m_{1}\left(A_{i}\right)+m_{2}\left(A_{i}\right)+\cdots +m_{n}\left(A_{i}\right)\right). \end{array}$$

In order to describe and evaluate the relationship between evidences in multiple dimensions, some research scholars calculate the degree of similarity between evidences by designing functions and put forward the concept of evidence distance. Generally speaking, the greater the degree of similarity between *m*_*n*_(*A*_*i*_) evidence, the smaller the distance of evidence. On the contrary, the smaller the degree of similarity between two pieces of evidence, the greater the distance between the evidence.

Assuming that *m*_1_ and *m*_2_ are the basic reliability functions of the evidence, the evidence distance between the evidences can be expressed as

(6) $$\begin{array}{c} d_{ij}=\sqrt{\frac{1}{2}\left({\left\|m_{i}\right\|}^{2}+{\left\|m_{j}\right\|}^{2}-2\langle m_{i},m_{j}\rangle \right)}. \end{array}$$

It is difficult to obtain the basic reliability function, and there is no unified solution in actual application. When the amount of evidence increases, the calculation of evidence theory may explode exponentially. The most prominent one is the failure of fusion when the evidence theory synthesizes conflicting evidence. The improved evidence algorithm effectively solves this problem [24].

### 2.2. Support Vector Machine Algorithm

Support vector machine, also known as “support vector network,” is a discriminative machine learning classification algorithm. It uses decision boundaries (hyperplanes in this case) to separate data points into two classes at a time. Support vector machine (SVM) classification is based on the principle of structural risk minimization. Seek an optimal hyperplane, which maximizes the blank area on both sides of the hyperplane while ensuring the classification accuracy of the training samples [25]. For the linear case, support vector machine is shown in Figure 4.

As shown in Figure 4, straight line *D* is a dividing line with *w* as the normal vector, which can divide the two types of data as accurately as possible. *D*2 is the support vector point in the two types of samples and is a straight line parallel to the classification line. When *D* is in the middle, the straight line satisfies the principle of maximizing the interval between the two types of sample points and becomes the optimal dividing line, which is transformed into the problem of finding the normal vector *w*. Extending to a high-dimensional space, the optimal classification line becomes the optimal hyperplane, that is, finding the normal vector of the optimal classification hyperplane, and classifying multiclass samples by finding the distance [26].

Taking the two-classification problem as an example, given the training sample set (*a*_*i*_, *b*_*i*_) of two types of data. In order to enable the hyperplane to correctly classify the two types of samples and to make the classification interval as large as possible, the hyperplane must satisfy

(7) $$\begin{array}{c} w\cdot a_{i}+b\geq 1. \end{array}$$

Then, the classification interval can be expressed as

(8) $$\begin{array}{c} \min\Phi \left(w\right)=\frac{1}{2}{\left\|w\right\|}^{2}=\frac{1}{2}\left(w^{t}\cdot w\right). \end{array}$$

When there is a linear inseparable pattern, the optimal segmentation hyperplane is required to meet the principle of minimum average classification error probability for all training samples. At this time, only the constraint condition of equation (8) is relaxed; that is, a slack variable *ξ*_*i*_ ≥ 0 is introduced, and then equation (8) becomes

(9) $$\begin{array}{c} b_{i}\left(w\cdot a_{i}+b\right)\geq 1-\xi_{i},\;i=1,2,\ldots ,n. \end{array}$$

This is to introduce a cost function into the objective function; that is, add a penalty component with an adjustable factor *C* to the function. So the objective function is

(10) $$\begin{array}{c} \min\Phi \left(w\right)=\frac{1}{2}{\left\|w\right\|}^{2}+c\sum_{i=1}^{n}\xi_{i}=\frac{1}{2}\left(w^{t}\cdot w\right)+c\sum_{i=1}^{n}\xi_{i}, \end{array}$$

where *c* is the penalty factor, which controls the degree of punishment for the wrong sample. The larger the *c*, the heavier the penalty for the error. In order to solve this constrained optimal problem, the Lagrange function is introduced. For the following equation,

(11) $$\begin{array}{c} L\left(w,x,y\right)=\frac{1}{2}{\left\|w\right\|}^{2}+c\sum_{i=1}^{n}\xi_{i}-\sum_{i=1}^{n}x_{i}\left(y_{i}\left(w\cdot x_{i}+y\right)-1\right). \end{array}$$

The Lagrangian function is only the function of conservative force in the mechanical system, and it is a function that describes the dynamic state of the whole physical system. Defined in analytical mechanics, the Lagrangian function of a dynamical system is a function that describes the dynamical state of the entire physical system. In the formula, *x*_*i*_ ≥ 0 is called the Lagrange (Lagrange) factor. The solution of the constrained optimization problem is determined by the saddle point of the Lagrange function. The solution of the optimization problem satisfies the partial derivative of *w* and *y* to be 0 at the saddle point. By seeking the partial derivative, the above problem is transformed into a simple dual problem, which is

(12) $$\begin{array}{c} \min\frac{1}{2}\sum_{j=1}^{n}\sum_{j=1}^{n}\alpha_{i}\alpha_{j}y_{i}y_{j}-\sum_{i=1}^{n}\alpha_{i}. \end{array}$$

For nonlinear classification problems, the sample can be projected to a high-dimensional space through an unknown mapping. The kernel function is the support vector machine that maps the input space to the high-dimensional feature space through a nonlinear transformation. The dimensionality of the feature space can be very high. If the solution of the support vector machine only uses the inner product operation, and there is a function in the low-dimensional input space, it is exactly equal to the inner product in the high-dimensional space. This mapping can be solved by using a kernel function. All functions that satisfy Mercer's theorem can be used as kernel functions, so that support vector machines can solve nonlinear problems in linear mode [27]. By constructing the optimization problem, only the inner product between samples appears in the solution process and in the final model. Therefore, when modeling nonlinear models, first defining the kernel function can solve the problem of unknown high-dimensional space mapping [28].

The kernel function method performs nonlinear classification, and the computational complexity of the algorithm itself does not increase. At this time, the dual problem can be expressed as

(13) $$\begin{array}{c} \sum_{i=1}^{n}\alpha_{i}b_{i}=0, \end{array}$$

where *α*_*i*_ is the Lagrangian factor and *b*_*i*_ is the number of support vectors.

It can be seen from equation (13) that for two classification problems, the algorithm seeks two hyperplanes, and each hyperplane corresponds to a class of samples. In the classification test, the distance between the data and the hyperplane is calculated, and the sample is classified into the category represented by the closer plane. In other words, Gemini Support Vector Machine contains one-to-two planning problems, each object function corresponds to one type of sample, and the constraint conditions are determined by the characteristics of another type of sample [29].

### 2.3. Taxonomy Based on Data Mining

Data mining refers to the process of searching for information hidden in a large amount of data through algorithms [30–32]. Data mining is usually related to computer science and achieves the above goals through a number of methods such as statistics, online analytical processing, intelligence retrieval, machine learning, expert systems, and pattern recognition. Classification plays an extremely important role in the field of data mining, analyzing data to extract data class models. This described model is called a classifier, which is specifically used to predict the class of data classification and give a unique class identification number. Classification technology can distinguish categories from samples of unknown categories, so as to provide a powerful reference for decision-making. Therefore, classification technology is widely used in systems with diagnostic and rating functions.

Suppose *S* is a set of data samples, the capacity is set to *a*, *m* different types of *C*, *a*_*i*_ is the number of samples of *C*_*i*_, *P*_*i*_ is the probability of any sample belonging to *C*_*i*_, and then, the entropy required for the classification of a given sample is

(14) $$\begin{array}{c} \text{Entropy}\left(a_{1},a_{2},\ldots ,a_{m}\right)=-\sum_{i=1}^{m}p_{i}\log_{2}\left(p_{i}\right). \end{array}$$

Suppose the value set of noncategory attribute *A* is (*a*_*ij*_,…, *a*_*mj*_), divide *A* into *v* subsets (*a*_1_,…, *a*_*N*_), where *a*_*j*_ is the sample on *A* and *a*_*ij*_ is the number of samples of *C*_*i*_ in *a*_*j*_, and the entropy is

(15) $$\begin{array}{c} \text{Entropy}\left(\text{A}\right)=-\sum_{i=1}^{m}\frac{a_{1j}+\cdots +a_{mj}}{a}\text{Entropy}\left(a_{ij},\text{…},a_{mj}\right). \end{array}$$

The information gain ratio is defined as

(16) $$\begin{array}{c} \text{Gainratio}\left(A,B\right)=\frac{\text{Gain}\left(A,B\right)}{\text{Split information}\left(A,B\right)}, \end{array}$$

where Gainratio(*A*, *B*) is the information gain, defined as

(17) $$\begin{array}{c} \text{Gainratio}\left(A,B\right)=\text{Entropy}\left(a_{1},a_{2},\ldots ,a_{m}\right)-\text{Entropy}\left(A\right). \end{array}$$

Split information(*A*, *B*) is the split information, which indicates the uniformity of the attribute split data, which is

(18) $$\begin{array}{c} \text{Split information}\left(A,B\right)=-\sum_{I=1}^{C}\frac{\left|A_{1}\right|}{\left|A\right|}\log_{2}\frac{\left|A_{i}\right|}{\left|A\right|}. \end{array}$$

It is used to evaluate whether a classification model prediction is accurate, and the most recognized index by the industry is to consider the recall rate and the correct rate. The ratio of the number of correctly classified positives to the actual total number of positives is called the recall rate, which is

(19) $$\begin{array}{c} \text{Recall}=\frac{\text{TP}}{P}. \end{array}$$

Recall is used to evaluate the reliability of the constructed classification model for the prediction of positive cases. In fact, in data research conducted in most engineering application environments, the attention paid to the positive target is far greater than the negative, so the recall rate is generally used as the most important indicator to measure the performance of the classifier. In addition, it is more intuitive that the concept of correct rate Accuracy is

(20) $$\begin{array}{c} \text{Accuracy}=\frac{\left(\text{TP}+\text{TN}\right)}{C}, \end{array}$$

where TP stands for true positive and TN stands for true negative.

In order to fully illustrate the advantages of the improved algorithm compared to other classification algorithms, the recall rate is used to conduct experimental comparisons under different scale datasets to verify the improved effect. Improved algorithm under different dataset sizes is Figure 5:

The recall rate is for the original sample, which indicates how many positive examples in the sample are predicted correctly. As shown in Figure 5, it can be seen that the improved classification algorithm has a higher recall rate regardless of whether it is under the small-scale dataset or under the condition of big data. When the dataset size is below 1300, the advantage is not big, but when the dataset size reaches 1400, it has obvious advantages, and the gap is very obvious under the data level after 1700. Combining with the foregoing, the improved algorithm is very suitable for the medical intelligent diagnosis and classification business in the era of big data.

## 3. Investigation, Experiment, and Analysis of Factors and Measures for Athletes with Ankle Joint Injuries

### 3.1. Investigation and Analysis of Factors and Types of Ankle Injuries

Ankle injury is the most common sports injury in sports. Athletes' own technology, quality, self-defense awareness, etc. will cause varying degrees of injury and will inevitably cause mild or severe sports injuries. This not only damages the health and athletic ability of the enthusiasts, but also has a negative impact on daily life, study, and physical exercise. This will bring various psychological barriers to the athletes and affect their enthusiasm for participating in sports training.

In this article, the injury site is divided into the lateral malleolus, medial malleolus, ankle heel, and foot on the side of the dominant foot and the nondominant foot side according to the original location of the pain. Types of injuries on the side of the dominant foot are shown in Tables 1 and 2.

From the comparison of Tables 1 and 2, it can be seen that athletes' feet injured mainly include the outer ankle, the inner ankle, the heel, and the ankle heel. The number of ligament strains on the dominant foot of athletes is the largest, with 105, and the number of ligament strains on the nondominant foot is 87. This shows that the athlete's dominant foot is more likely to be injured than the nondominant foot.

This article investigates the proportion of athletes' ankle injuries in 2019 and 2020, as shown in Figure 6.

The percentage of athletes with ankle injuries in 2019 started at about 10%. Although it declined later, it has been on an upward trend, rising to about 25%; the percentage in 2020 has risen from about 13% at the beginning to the best 33% of the total, which is faster than the increase in 2019. As shown in Figure 6, from 2019 to 2020, the proportion of athletes' ankle injuries is increasing. Ankle injuries are mostly caused by indirect external forces. The components of the ankle joint are photographed as physical damage, so that the ankle joint cannot be extended, rotated, and rotated normally. If it is not treated in time or treatment is not thorough, it will affect the ability of the ankle joint in the future.

This article divides the injuries of 100 sports personnel into 2 levels, as shown in Table 3.

As shown in Table 3, sports injuries can be simply divided into two levels. The first levelincludes acute injury and chronic injury. Among them, the number of acutely injured is 75, accounting for 75%; the number of chronically injured is 25, accounting for 25%. It can be seen that acute injury is much higher than chronic injury.

Among them, the secondary injury of acute injury includes the following points, as shown in Table 4.

Among them, the number of ankle injuries is the largest, with 25 people, accounting for 33%, the highest proportion. It can be seen from Table 4 that acute secondary injuries include ankle injuries, bruises, sprains, and strains. Among them, the proportion of ankle joint injuries is the highest. Because sports is a physical antagonistic sport, it has the characteristics of small playing field, fast offensive and defensive conversion, fierce competition, and strong physical antagonism. The athletes have poor self-protection consciousness. They can't pay attention to the control of their own movements during exercise, and often do quick and acute movements, which are more prone to ankle sprains, bruises, and contusions.

In order to verify the reliability of the data, this article conducted a survey of the types of injuries in the sports majors of 6 universities, as shown in Figure 7.

As shown in Figure 7, the injury sites of sports majors in 6 colleges and universities mainly include ankle joint injury, knee joint injury, thigh injury, calf injury, upper limb, and head injury. Among them, the proportion of ankle joint injuries is the highest, and the proportion range is 54%–70%. It can be seen that ankle joint injuries should be paid attention to.

In order to make the results of the experiment clearer, this article investigates the injury factors of sports players, as shown in Table 5.

As shown in Table 5, the main factors for athletes' injuries include incorrect technique, poor awareness of protection, overburdened ankle joints, other reasons, and poor physical fitness. Among them, the score of technically incorrect is 67 points, accounting for 32.5%, ranking first. The score for poor protection awareness is 35 points.

This article investigates the main injury factors of athletes from 2016 to 2020, as shown in Figure 8.

As shown in Figure 8, the main causes of injuries for athletes from 2016 to 2020 include incorrect technique, poor protection awareness, overburdened ankle joints, other reasons, and poor physical fitness. Among them, the proportion of incorrect technology is the highest, rising from 8% in 2016 to 14% in 2020; the percentage of poor protection awareness has risen from 7% in 2016 to 13% in 2020. Among them, the percentage of incorrect technology is the highest, reaching 14% in 2020. Therefore, it is necessary to strengthen the study of professional technology.

In summary, the main causes of ankle joint injuries are as follows:

1. Incorrect technology
2. The criterion of whether the technology is reasonable is to meet the requirements of the laws of human motion mechanics and biology. Technology is the performance of a general law with commonality, but it is necessary to consider the commonalities and the characteristics of each athlete at the same time. The unity of individuality and commonality is the best technique. Special technology is the basis for special sports. Therefore, the correct technical actions must be ensured.
3. Poor protection awareness
4. Because sports is a combination of speed, endurance, strength, and skill, injuries are often accompanied by sports, and some injuries can be avoided by effective methods. The injury of the ankle joint happened suddenly and without warning, and only through the education of protective awareness and simulation measures to avoid the injury.
5. Overburden on the ankle joint
6. In sports, every movement is based on the ankle joint, which is the key point of the entire sports. In sports, the rapid turning, sudden stop, and sudden rise all cause strong pressure on the ankle joint. Relevant studies have shown that the supporting stage of running is twice the load of the joints when walking. The joints bearing such a large force must undergo special training to strengthen the ankle joint's ability to bear the force.
7. Other reasons
8. The remaining items include three factors: venue and equipment problems, clothing and shoes problems, and insufficient preparation activities. On the surface, these three factors are not related to ankle joint injury, but it is found through investigation that they are one of the main factors of sports ankle joint injury.

### 3.2. Experiment and Analysis of Comprehensive Rehabilitation Nursing for Ankle Joint Injury Rehabilitation

Nowadays, due to various reasons such as the aging of the city and the complexity of urban traffic, ankle joint fractures account for an increasing proportion of the whole body fractures, and they have become one of the most common fractures in trauma orthopedics clinics. Ankle fractures caused by sports can account for about 7% of ankle fractures, which have an important impact on the life of patients and the development of society. Since sports ankle fractures are intra-articular fractures, this has higher requirements for surgery. Anatomical reduction must be given to avoid serious complications such as traumatic arthritis as much as possible.

This requires targeted guidance of patients to carry out early rehabilitation exercises in order to restore the patients' normal physiological functions as much as possible. This article compares the recovery speed of ankle joint injuries before and after rehabilitation care, as shown in Table 6.

As shown in Table 6, the recovery speed of patients who underwent comprehensive rehabilitation care was significantly higher than that before recovery care. It can be seen that comprehensive rehabilitation care is of great importance to the degree of recovery of patients, and rehabilitation care is also necessary.

#### 3.2.1. Establish the Concept and Awareness of Early Rehabilitation

Rehabilitation of bone and joint injuries must be emphasized as early as possible, and interventional rehabilitation work should be carried out as soon as the patient's general condition permits. It creates favorable conditions for later functional recovery, actively prevents and reduces the occurrence of related complications, and must not separate treatment and rehabilitation. Those who think that after the treatment is over, the actions of the doctors who perform rehabilitation are even more inappropriate, which will be extremely unfavorable to the patient's functional recovery. Therefore, early functional exercise must be carried out.

#### 3.2.2. “Combination of Dynamic and Static”

Combination of fixation and exercise: After the fracture is reliably fixed by the operation, guided functional rehabilitation exercise is performed when the patient's pain is relieved, so as to restore the patient's normal physiological function as soon as possible. It is in the principle of fracture treatment of “combination of movement and static, equal emphasis on muscles and bones” in Chinese medicine. “Static” refers to the reliable fixation of fractures, including internal fixation and external fixation, while “movement” refers to functional exercise activities carried out under reliable fixation. “Dynamic” and “static” are inextricably related to each other. Functional exercise after fracture needs to be carried out under reliable fixation and does not affect fracture healing. The purpose of fracture fixation is to restore the patient's physiological function as much as possible. This kind of rehabilitation exercise method has great advantages and feasibility. It is a trustworthy, safe, and effective rehabilitation method.

## 4. Discussion

This article analyzes how to analyze the impact of comprehensive rehabilitation nursing on the rehabilitation of sports-induced ankle injuries based on the smart medical system. It expounds the concepts related to smart medical care and ankle joint injuries, and studies algorithms based on data mining and related theories of comprehensive rehabilitation care. It also explored how to prevent ankle joint injuries caused by exercise, and through experiments to discuss the importance of comprehensive rehabilitation care for the recovery of ankle joint injuries caused by exercise.

This article also makes reasonable use of data mining methods based on smart medical care. As the scope of application of data mining methods has become larger and larger, the importance has also increased. According to this calculation, it is very important to discover the importance of comprehensive rehabilitation nursing for the recovery of ankle joint injuries caused by exercise based on data mining.

Through the experiments of many sports athletes, this article shows that with the development of the sports field in recent years, people are more and more likely to be injured in sports. Among them, ankle joint injury is a relatively common injury. There are many factors for ankle injury, such as insufficient professional skills, and weaker body, which requires athletes to improve their professional capabilities.

## 5. Conclusions

This article mainly discusses the effect of comprehensive rehabilitation nursing on the rehabilitation of sports-induced ankle joint injuries. This article adds an introduction to smart medical care. Based on smart medical care, it proposes a multisource data fusion and a classification method based on data mining and expounds the concepts of smart medical care and comprehensive rehabilitation care. The two algorithms are also specifically introduced in the method section. In the experimental part, a number of sports athletes in a number of universities were investigated, and it was found that the current ankle joint injury is one of the more frequent sports injuries. Through the comparison before and after rehabilitation care, it is found that comprehensive rehabilitation care plays a better role in the recovery speed of patients. The injury of the ankle joint will not only have a serious impact on the athlete's athletic ability, but also cause certain harm to the athlete's healthy development. If effective countermeasures are not taken to prevent sports injuries, it will have a serious adverse effect on the promotion and development of sports. Therefore, it is very important to analyze the causes of sports ankle joint injuries and propose comprehensive rehabilitation nursing measures.

## Figures and Tables

**Figure 1:** Simulated ankle injury.

**Figure 2:** The structure of multisource data fusion.

**Figure 3:** Fusion computing.

**Figure 4:** Support vector machine.

**Figure 5:** Improved algorithm under different data set sizes.

**Figure 6:** Proportion of athletes with ankle injuries in 2019 and 2020. (a) Proportion of athletes with ankle injuries in 2019. (b) Proportion of athletes with ankle injuries in 2020.

**Figure 7:** 6 injury types of sports professional athletes in colleges and universities.

**Figure 8:** Major injury factors for athletes from 2016 to 2020.

**Table 1:** Types of injuries on the side of the dominant foot.

Dominant foot	Ligament strain	Inflammation of the tendon	Fracture
Lateral malleolus	105	43	4
Medial malleolus	32	20	3
Ankle heel	15	5	2
Heel	10	2	0

**Table 2:** Types of nondominant foot side injuries.

Nondominant foot	Ligament strain	Inflammation of the tendon	Fracture
Lateral malleolus	87	35	2
Medial malleolus	25	15	0
Ankle heel	10	4	0
Heel	5	1	0

**Table 3:** Acute injury primary injury questionnaire.

First degree injury	Number of people	Percentage (%)
Acute injury	75	75
Chronic injury	25	25
Total	100	100

**Table 4:** Acute injury secondary injury questionnaire.

Secondary damage	Number of people	Percentage (%)
Ankle injury	25	33
Sprain	18	24
Strain	17	22
Bruise	15	21
Total	75	100

**Table 5:** Injury factors of sports players.

Sort	Injury factor	Score	Percentage (%)
1	Incorrect technique	67	32.5
2	Poor protection awareness	54	26.2
3	Overburdened ankle	35	20
4	Other reasons	30	11.3
5	Poor physical fitness	20	10

**Table 6:** Recovery speed of ankle joint injury before and after rehabilitation care.

Object	After care (%)	Before care (%)
1	20	14
2	25	12
3	19	8
4	17	9
5	27	10

## Data Availability

No data were used to support this study.
